This article has been retracted.

# What Promotes Medical Overuse: Perspective on Evolutionary Game between Administration and Medical Institutions

**DOI:** 10.1155/2022/4351282

**Published:** 2022-09-14

**Authors:** Chenxi Xu, Li Luo, Siyu Zeng, Xiaozhou He, Jialing Li, Guiju Zhu

**Affiliations:** ^1^Business School, Sichuan University, No. 24 South Section 1, Yihuan Road, Chengdu, China; ^2^School of Logistics, Chengdu University of Information Technology, No. 10, Xingfu Road, Chengdu, China; ^3^School of Management, Hunan University of Technology and Business, No. 569 Yuelu Avenue, Changsha, China

## Abstract

Medical overuse is the leading cause of high expenditure among healthcare systems worldwide, with the degree varying from region to region. There is increasing evidence to indicate that in China, National Healthcare Security Administration (NHSA) supervision plays the most crucial role in decreasing medical overuse. For medical overuse, traditional studies focus on empirical researches and qualitative analysis, most of which ignore how the two important participants, i.e., medical institutions and NHSA, affect the strategy of each other. To reduce the losses incurred by insufficient supervision, this study starts from bounded rationality, builds an evolutionary game model to study the relations between the NHSA and medical institutions, and reveals the dynamic evolution process of the supervision of NHSA and overuse of medical institutions. Through stable evolutionary strategy analysis, numerical simulation results, and sensitive experiments under diverse scenarios, we found that when profit gap of medical overuse is high or low, medical institution will adopt fixed strategy, which is medical overuse or appropriate medical use. Only when the profit gap is at a medium level will NHSA's choice affects medical institutions' strategy. Furthermore, NHSA's strategy is affected by the profit gap between medical use and supervision cost. Our work enriches the understanding of supervision for medical overuse and provides theoretical support for the NHSA to make decisions to reach an ideal condition, i.e., to supervise without exertion.

## 1. Introduction

Medical overuse is defined as the provision of superfluous healthcare services. It involves the unnecessary expenditure of resources beyond the actual needs of a medical condition, which might even result in possible harm [1–3].

Medical overuse is the leading cause of high expenditure among healthcare systems worldwide [4, 5]. Previous studies have estimated that approximately 30% of healthcare spending might be considered wasted expenditure [6]. In the United States, waste from overuse costs more than $210 billion a year [7], and this figure is even higher in low- and middle-income countries [3]. Elimination of medical overuse could substantially improve healthcare efficiency. The reasons that lead to medical overuse are complex, such as insufficient investment by the government, the pharmaceutical industry's incentives to doctors, hospitals' pursuit of increased profits, and patients' demand for additional medical services to promote faster recovery [8]. Furthermore, the information asymmetry between doctors, patients, and insurance companies leads to considerable risks and uncertainty in the purchase of medical services, which leads to excessive medical treatment [9]. The Chinese medical care system has experienced noteworthy changes after three decades of reform, which improved medical insurance coverage [10]. Most medical expenditure is paid for by the National Healthcare Security Administration (NHSA) in China, but the NHSA is facing a serious imbalance of income and expenditure and continuous growth of medical expenses [11]. In China, the current medical insurance payment is mostly based on fee-for-service; that is, the insurer compensates according to the quantity and price of medical services provided in a certain proportion. This payment method makes hospitals hardly bear the risk of rising medical costs and obtain higher income by increasing the number of medical services. Therefore, hospitals not only lack initiative to control medical costs but also induce demand and provide unnecessary medical services, which is medical overuse [12]. China is at a loss as to how to transform its new money into efficient and effective healthcare. Many papers argue that unless China tackles the root causes of wasteful healthcare delivery, the healthcare system will be severely threatened [13]. Thus, reducing medical overuse is an urgent concern for the Chinese government.

As a result, many studies focused on understanding how to mitigate medical overuse [1]. Previous studies mainly focused on retrospective analysis of data [14, 15] or on the analysis of treatment for a specific disease or the overuse of a single service [16] and the influence factors of medical overuse [17, 18]; some findings sought to determine if there was variance among medical specialties [19]. To reduce medical overuse, it is found that intervention's impact on media coverage of medicine can help patients to stay away from medical overuse [20]. It is found that NHSA's supervising and punishment of doctors' behaviour, establishing reputation mechanism, and protecting patient's right are important factors to restrain medical overuse behaviour [21]. Most of them suggested that strengthening NHSA's supervision could decrease the overuse of medical service [22] but did not make detailed suggestions regarding ways to regulate it. Previous studies tend to start from a single perspective, but there is still a lack of research on the evolutionary game in which NHSA and medical institutions are fully integrated under the background of FFS (fee-for-service).

In this study, however, we aim at figuring out the interest coordination of the main stakeholders in medical overuse based on evolutionary game theory whose formation and evolution is an interactive and game process between the two organisations, that is, NHSA and medical institutions. And we construct a dynamic evolutionary game model to investigate the supervisory mechanism for reducing medical overuse in government and hospitals, based on the premise of limited rationality. With the constructed model, we first analyse evolutionary stable strategies and then make further analysis on equilibrium stable strategy. And via numerical simulation on MATLAB with the model and stable strategies, we explore what factors influence the strategy making of medical institutions and NHSA.

To build the evolutionary game model, we first need to make clear the game mechanism. So, what is the NHSA's regulatory mechanism for medical institutions on medical overuse? NHSA and medical institutions are two participants in the decision-making of reducing medical overuse. For NHSA, the strategies are composed of strict supervision and loose supervision. And for medical institutions, the strategies are composed of medical overuse and appropriate medical overuse. For the two participants, different strategies will lead to different profit and cost, which will also affect the decision-making of both sides. The hardcore is to dig out how the variation of cost and profit is related to the strategy adoption of NHSA and medical institutions.

This paper discusses the influence of the profit gap between medical overuse and appropriate use and supervision costs on the decision-making of NHSA and medical institutions by analysing six scenarios. There are two main contributions:

1. A model based on game theory is proposed to design mechanism and solve issues on overuse medical costs via analysing the strategies between medical institutions and NHSA with the consideration of patient supervision
2. The proposed model and the numerical experiments under different scenarios show the factors influencing decision-making of NHSA and medical institutions and suggest that to reduce the occurrence of medical overuse, this paper finds that minimizing the high profits of medical overuse from the source forward is more effective than to strengthen supervision

This paper is organised as follows: Section 2 is the literature review; Section 3 describes the construction of an evolutionary game model and discussion of the equilibrium of the model; Section 4 explains the simulation analysis of the game model; and Section 5 presents the results and conclusions.

## 2. Literature Review

### 2.1. Effect of Medical Overuse

Scholars conducted extensive studies to explore the reason of the continuous increase of medical cost. Worldwide, the growth in healthcare expenditure from the rising volume of medical services has been identified as the biggest threat to government finances. Population growth and ageing are believed to be the leading causes of medical cost increase over last century [23]. Recently, Berwick and Andrew [24] and Daley and Savage [25] suggested another root cause: medical overuse. Wennberg et al. indicated that the proportion of Medicare spending owing to overuse is almost 29% [26]. Korenstein et al. claimed that overuse can be as high as 89% in certain populations worldwide [27]. A study published in Lancet in 2007 pointed out that overuse is harmful to patients and healthcare systems, and thus, physicians, politicians, and policy-makers must understand overuse and act to reduce it [3]. These studies suggested that medical overuse is the main reason of high medical expenditure.

Medical overuse will not only increase medical costs but also do harm to patients' health. The risk of harm from overuse varies depending on the disease [28]. Bansal et al. discussed end-of-life medication for cancer patients, half of whom received ineffective radiotherapy [16]. Ming et al. reviewed the situation, reasons, and countermeasures of overuse of cardiovascular services in America and explored its implications to China [22]. Researchers are also concerned about the overuse of certain medical services. The use of antibiotics, which is a global overuse problem, has drawn considerable attention [14]. André et al. [15], Gulliford et al. [29], and Panasiuk et al. [30] proved that 50% of patients receive unnecessary antibiotics. Currie et al. tested antibiotics abuse in China [31]. Xiang and Yan analysed the overuse of injections in China [32]. Taasan and Winchester used patients' hospitalisation data between 2012 and 2015 to identify the overuse of cardiac troponin [33]. Romano et al. [34] evaluated continuity using the Bice–Boxerman continuity of care index and discovered that higher continuity of care could reduce medical overuse. All of these studies point out the harm of medical overuse and the need to decrease it.

### 2.2. Reasons of Medical Overuse

Lots of studies focus on how to reduce medical overuse. A few papers suggested strategies to mitigate overuse, and monitoring is seen to be one of the most effective measures [22, 35]. Supervision of medical overuse generally considers three aspects: internal supervision of hospitals [22], patients [36], and government departments [22]. McCulloch et al. pointed out that interventions targeting healthcare systems using financial, regulatory, or incentivisation strategies may reduce overuse of surgery [35]. Arab-Zozani et al. [36] and McCulloch et al. [35] suggested that patient engagement, such as shared decision-making, may reduce medical overuse. Ming et al. suggested that strengthening government supervision could decrease the overuse of medical services [22]. A few studies considered the supervision of medical institutions by both patients and NHSA. However, none of these studies analysed how NHSA regulations to supervise medical costs can affect the strategy selection of hospitals, which in turn affects the use of insurance funds. Furthermore, few studies have considered the impact of patient complaints. We aim to address these lacunae in our research.

### 2.3. Applications of Evolutionary Game Theory

Scholars' applications of evolutionary game theory among stakeholders bring inspirations to this study. Evolutionary game theory is a successful mathematical framework geared towards understanding the selections that affect the evolution of the strategies of agents engaged in interactions with potential conflicts [37], fully take into account the behaviours of multiple participants, and analyse the interaction of behavioural changes of participants dynamically. It considers the bounded rationality of the decision-maker and is widely used in many fields [38]. Chen et al. built an evolutionary game model to consider green retrofitting from the perspective of green credit [39]. Yang used an evolutionary game to analyse the cooperative construction of international transport corridors [40]. Wu et al. built a complex model of an evolutionary game between the government and enterprises in a low-carbon network environment and studied the effect of government incentives for enterprises [41]. Luo and Zhao used an evolutionary game to find ways to reduce food waste [42]. It is a good tool to fulfill the expectation of maximizing stakeholder interests by predicting the behaviour of others to determine the most advantageous strategy [43].

### 2.4. Summary

In sum, an evolutionary game is an effective way to explore the regulatory mechanism of NHSA to reduce medical overuse, but the existing research focuses on using historical data to analyse the medical overuse from doctors or opinions from the perspective of NHSA's supervision. Therefore, we proposed an evolutionary game theory to construct a dynamic evolutionary game model between hospitals' medical overuse and NHSA supervision. We also considered patients' complaints as third-party supervision to investigate the supervisory mechanism for reducing medical overuse in the NHSA and hospitals. From the perspective of NHSA supervision, we explore the punishment-and-reward mechanism to ensure the stability of both sides. We also summarise countermeasures and suggestions conducive to reducing excessive medical treatment, to enable the medical insurance fund to play a better role.

## 3. Evolutionary Game Model

### 3.1. Problem Description

Medical overuse has increasingly attracted the attentions and discussions in the academic field. On the one hand, the NHSA's lack of professionalism makes it difficult to review the reasonableness of diagnosis and treatment, and hence, its supervision is insufficient [44]. In order to maximize the income, the hospital will increase the income of nondrug medical services through too many examinations and tests. On the other hand, the total revenue of the hospital can be expanded by allowing patients to make multiple visits [45]. The patient had less health-related knowledge, and misconception of medical overuse, doctor-patient communication, and information asymmetry will affect patients' medical overuse cognition, eventually leading to their overtreatment behavioural choices [46]. In summary, policy-makers are faced with the challenge of how to urge medical overuse. Thus, in order to comprehensively explore the relationship between NHSA and medical institutions, an evolutionary game model is developed.

#### 3.1.1. Basic Assumption

Medical insurance departments and medical institutions face a very complex decision-making environment in attempting to reduce medical overuse. Therefore, for the convenience of analysis, some basic assumptions are set in advance as follows.

*(1) Only Two Parties in the Game*. NHSA and medical institutions are the two participants in the game model, and they are all bounded rational.

In this study, we assumed the relationship between doctors and medical institutions is a traditional principal-agent relationship; i.e., the behaviour of doctors is consistent with that of medical institutions [47].

*(2) Behaviour Strategies*. There are two kinds of supervision strategies that NHSA can offer, i.e., strict and loose. Strict supervision generally means that the NHSA will expend considerable money, time, and human resources to regulate doctors' behaviour, by means such as increasing the frequency of spot checks and appointing inspectors. Loose supervision implies that the NHSA will not take additional restrictive measures but conduct some routine inspections and so on. Medical institutions also have two kinds of strategies, i.e., medical overuse and appropriate medical use. Appropriate medical use means that the doctor will make a diagnosis and treatment plan that is most suitable for the patient according to the patient's condition. Conversely, medical overuse refers to doctors tending to provide excessive medical treatment to get extra benefits, such as some unnecessary drug prescriptions and medical examination.

#### 3.1.2. Parameter Assumption

*(1) Assumption 1*. Assume that NHSA offers “strict supervision” at a rate of *p* and “loose supervision” at a rate of 1 − *p*; assume that medical institutions choose “appropriate medical use” at a rate of *q* and choose “medical overuse” at a rate of 1 − *q*, where *p*, *q* ∈ [0, 1].

*(2) Assumption 2*. The cost of NHSA is *C*_1_ when it offers strict supervision and 0 when it offers loose supervision. Under strict supervision, the administration can detect medical overuse behaviour before patients.

*(3) Assumption 3*. If and when the medical institution's excessive diagnosis and treatment behaviour is discovered, the NHSA will impose a penalty of *F* upon the medical institution, which will cause the hospital to incur a reputation loss of *M*.

*(4) Assumption 4*. The marginal revenue of appropriate medical use in medical institutions is *R*_1_, and the marginal revenue of medical overuse is *R*_2_, with *R*_1_ < *R*_2_. The profit gap is then denoted as ∆*R* = *R*_2_ − *R*_1_. Appropriate medical use behaviours of medical institutions can also improve an institution's reputation, attracting more patients, and the revenue associated with reputation is *R*_3_.

*(5) Assumption 5*. Under loose supervision, patients will question the medical overuse behaviour of medical institutions and have a probability of *θ* (0 < *θ* < 1) of reporting it to the NHSA.

*(6) Assumption 6*. After the patients' reporting to NHSA, the administration needs to conduct further verification, which would cause reputation loss, and the cost of verification and loss are recorded as *C*_2_. The model parameters are summarised in Table 1, and the payoff matrix of the evolutionary game is displayed in Table 2.

### 3.2. Analysis of Evolutionary Stable Strategies

Variable *G*_1_ represents the expected payoff of NHSA when choosing the “strict supervision” strategy, while *G*_2_ represents the expected payoff of NHSA when choosing the “loose supervision” strategy, and $\bar{G}$ represents the average expected payoff. According to the assumptions and Tables 1 and 2, *G*_1_, *G*_2_, and $\bar{G}$ are as follows:

(1) $$\begin{array}{c} G_{1}=\left(-C_{1}+F\right)-qF, \end{array}$$

(2) $$\begin{array}{c} G_{2}=\theta \left(1-q\right)\left(F-C_{2}\right), \end{array}$$

(3) $$\begin{array}{c} \bar{G}={pG}_{1}+\left(1-p\right)G_{2}. \end{array}$$

Similarly, variable *E*_1_ represents the expected payoff of medical institutions when choosing the “appropriate medical use” strategy, *E*_2_ represents the expected payoff of medical institutions when choosing the “medical overuse” strategy, and $\bar{E}$ represents the average expected payoff. According to the assumptions and Tables 1 and 2, *E*_1_, *E*_2_, and $\bar{E}$ are as follows:

(4) $$\begin{array}{c} E_{1}={pR}_{3}+R_{1}, \end{array}$$

(5) $$\begin{array}{c} E_{2}=-p\left(1-\theta \right)\left(F+M\right)+\left[R_{2}-\theta \left(F+M\right)\right], \end{array}$$

(6) $$\begin{array}{c} \bar{E}={qE}_{1}+\left(1-q\right)E_{2}. \end{array}$$

Based on the principles of evolutionary games, the game dynamic replication equations between medical institutions and NHSA are as follows [48]:

(7) $$\begin{array}{c} \left\{\begin{array}{c} F\left(p\right)=\frac{dp}{dt}=p\left(G_{1}-\bar{G}\right)=p\left(1-p\right)\left\{\left(1-q\right)\left[\left(1-\theta \right)F+\theta C_{2}\right]-C_{1}\right\},\\ F\left(q\right)=\frac{dq}{dt}=q\left(E_{1}-\bar{E}\right)=q\left(1-q\right)\left\{p\left[R_{3}+\left(1-\theta \right)\left(F+M\right)\right]+\left[R_{1}-R_{2}+\theta \left(F+M\right)\right]\right\}. \end{array}\right. \end{array}$$

The derivatives with respect to *F*(*p*) and *F*(*q*) are as follows:

(8) $$\begin{array}{c} \left\{\begin{array}{c} \frac{dF\left(p\right)}{dp}=\left(1-2p\right)\left\{\left(1-q\right)\left[\left(1-\theta \right)F+\theta C_{2}\right]-C_{1}\right\},\\ \frac{dF\left(q\right)}{dq}=\left(1-2q\right)\left\{p\left[R_{3}+\left(1-\theta \right)\left(F+M\right)\right]+\left[R_{1}-R_{2}+\theta \left(F+M\right)\right]\right\}. \end{array}\right. \end{array}$$

According to the stability theorem of differential equations, the equilibrium points of the replicator dynamic equations presented by (7) should satisfy *F*(*p*) = *F*(*q*) = 0, and {(*p*, *q*)|0 ≤ *p*, *q* ≤ 1}. Apparently, (0,0), (0,1), (1,0), and (1,1) are the four fixed equilibrium points. For convenience, let *p*∗ = (*R*_2_ − *R*_1_ − *θ*(*F* + *M*))/(*R*_3_ + (1 − *θ*)(*F* + *M*)) and *q*∗ = ((1 − *θ*)*F* + *θC*_2_ − *C*_1_)/((1 − *θ*)*F* + *θC*_2_); then, (*p*^∗^, *q*^∗^) is also an equilibrium point when meeting the following conditions: 0 ≤ (*R*_2_ − *R*_1_ − *θ*(*F* + *M*))/(*R*_3_ + (1 − *θ*)(*F* + *M*)) ≤ 1 and 0 ≤ ((1 − *θ*)*F* + *θC*_2_ − *C*_1_)/((1 − *θ*)*F* + *θC*_2_) ≤ 1.

According to the method proposed by Friedman [49], the stability at the equilibrium point of the evolution system can be judged by the local stability of the Jacobian matrix of the entire system. The Jacobian matrix of this system made of (7) is as follows:

(9) $$\begin{array}{c} J=\left[\begin{array}{cc} \frac{\partial F\left(p\right)}{\partial p} & \frac{\partial F\left(p\right)}{\partial q}\\ \frac{\partial F\left(q\right)}{\partial p} & \frac{\partial F\left(q\right)}{\partial q} \end{array}\right]=\left[\begin{array}{cc} \left(1-2p\right)\left\{\left(1-q\right)\left[\left(1-\theta \right)F+\theta C_{2}\right]-C_{1}\right\} & -p\left(1-p\right)\left[\left(1-\theta \right)F+\theta C_{2}\right]\\ q\left(1-q\right)\left[R_{3}+\left(1-\theta \right)\left(F+M\right)\right] & \left(1-2q\right)\left\{p\left[R_{3}+\left(1-\theta \right)\left(F+M\right)\right]+\left[R_{1}-R_{2}+\theta \left(F+M\right)\right]\right\} \end{array}\right]. \end{array}$$

The local equilibrium points (LEP) of the replicated dynamic system are judged as an evolutionarily stable strategy (ESS) if it satisfies the following conditions: det *J* > 0 and trac *J* < 0, where det *J* and trac *J* denote the determinant and trace of *J*, respectively. Meanwhile, to resist disturbance in the stable state, the ESS must satisfy the conditions (*dF*(*p*))/*dp* < 0 and (*dF*(*q*))/*dq* < 0. det *J* and trac *J* for each LEP are presented in Table 3.

### 3.3. Stability Analysis of Equilibrium Point

Furthermore, the stability of equilibrium points in the government–enterprise evolutionary game system will be analysed according to various value ranges of parameters. The det *J* and trac *J* of every point's Jacobi matrix point are calculated, and its state is discussed.

Scenario 1: *R*_2_ − *R*_1_ < *θ*(*F* + *M*_1_), *C*_1_ > (1 − *θ*)*F* + *θC*_2_

At this point, there are four fixed equilibrium points of the evolutionary game dynamic replication equations, i.e., (0,0), (0,1), (1,0), and (1,1).

For the hospital, the gap between the excess profit obtained through medical overuse and the profit obtained by appropriate medical use is less than the expected fines and reputation loss caused by patient complaints reporting medical overuse. Therefore, hospitals are more likely to choose appropriate medical use, while NHSA has a probability of 1 − *θ* of being fined and incurring reputation loss from loose supervision, which is the cost of less-than-strict supervision. Therefore, NHSA tends to choose loose supervision. For Scenario 1, as presented in Table 4, point (0,1) is the ESS of the system, namely, {loose supervision, appropriate medical use}.

Scenario 2: *θ*(*F* + *M*) < *R*_2_ − *R*_1_ < *R*_3_ + *F* + *M*, *C*_1_ > (1 − *θ*)*F* + *θC*_2_

At this point, there are four fixed equilibrium points of the evolutionary game dynamic replication equations, which are (0,0), (0,1), (1,0), and (1,1).

For the hospital, the difference between the profit obtained by medical overuse and the profit obtained by appropriate medical use is less than the revenue caused by reputation, but higher than the fines and reputation loss caused by medical overuse reported via patient complaints. Under circumstances where the medical overuse strategy is more profitable, hospitals are more likely to use medical resources excessively. For NHSA, the cost caused by fines and reputation loss is less than strict supervision. NHSA is more likely to choose loose supervision. For Scenario 2, as presented in Table 4, point (0,0) is the ESS of the system, namely, {loose supervision, medical overuse}.

Scenario 3: *R*_2_ − *R*_1_ > *R*_3_ + *F* + *M*, *C*_1_ > (1 − *θ*)*F* + *θC*_2_

At this point, there are four fixed equilibrium points of the evolutionary game dynamic replication equations, which are (0,0), (0,1), (1,0), and (1,1).

For the hospital, the difference between the profit obtained through medical overuse and the profit obtained by appropriate medical use is higher than the sum of reputation earnings by appropriate medical use and the fines and reputation loss caused by medical overuse. Under such circumstances, where the medical overuse strategy is more profitable, hospitals are more likely to choose excessive treatments. However, there is probability of 1 − *θ* that NHSA will fine them and they will suffer a loss of reputation under loose supervision. The high cost of strict supervision enforces the administration to choose the loose strategy. For Scenario 3, as presented in Table 4, point (0,0) is the ESS of the system, namely, {loose supervision, medical overuse}.

Scenario 4: *R*_2_ − *R*_1_ < *θ*(*F* + *M*), *C*_1_ < (1 − *θ*)*F* + *θC*_2_

At this point, there are four fixed equilibrium points of the evolutionary game dynamic replication equations, i.e., (0,0), (0,1), (1,0), and (1,1).

For the hospital, the difference between the profit obtained by medical overuse and the profit obtained by moderate treatment is less than the sum of reputation earnings by appropriate medical use and the fines and reputation loss caused by medical overuse. Without profits to earn, hospitals tend to adopt appropriate medical use. With fines and reputation loss at a probability of 1 − *θ* from loose supervision, NHSA tends to adopt strict supervision with a lower cost. For Scenario 4, as presented in Table 4, point (0,1) is the ESS of the system, namely, {loose supervision, appropriate medical use}.

Scenario 5: *θ*(*F* + *M*) < *R*_2_ − *R*_1_ < *R*_3_ + *F* + *M*, *C*_1_ < (1 − *θ*)*F* + *θC*_2_

At this point, there are five fixed equilibrium points of the evolutionary game dynamic replication equations, i.e., (0,0), (0,1), (1,0), (1,1), and (*p*^∗^,*q*^∗^).

For the hospital, the gap between the profit obtained by medical overuse and the profit obtained by appropriate medical use is less than the revenue associated with reputation, but higher than the fines and reputation loss caused by medical overuse. Under the circumstances, hospitals are more likely to use medical resources overly. However, for NHSA, the strict supervision is less than the cost caused by fines and reputation loss. NHSA is more likely to choose strict supervision. The strategy choices between the two sides are contradictory. For Scenario 5, as presented in Table 4, there is no ESS in the system; i.e., NHSA and medical institutions both choose a mixed strategy.

Scenario 6: *R*_2_ − *R*_1_ > *R*_3_ + *F* + *M*, *C*_1_ < (1 − *θ*)*F* + *θC*_2_

At this point, there are four fixed equilibrium points of the evolutionary game dynamic replication equations, i.e., (0,0), (0,1), (1,0), and (1,1).

For the hospital, the difference between the profit obtained by medical overuse and the profit obtained by appropriate medical use is not only higher than the revenue caused by reputation but also higher than the fines and reputation loss caused by medical overuse reported through patient complaints. With profits to earn, hospitals are more likely to choose overuse. The cost of fines and reputation loss from loose supervision is higher than that of strict supervision. Therefore, the administration tends to regulate strictly. For Scenario 6, as presented in Table 4, point (1,0) is the ESS of the system, namely, {strict supervision, medical overuse}.

In the study, we divide the profit gap into three levels, high, medium, and low, and divide the supervision cost into two levels, high and low, thus proposing six scenarios. Through the analysis above, the results corresponding to each scenario are listed in Table 5.

1. High profit gap

When the profits of medical overuse are high enough, medical institutions will choose medical overuse regardless of whether NHSA takes regulatory measures. For hospitals, the promotion of profit is far higher than the inhibition of supervision of NHSA. NHSA's choice of strategy totally depends on the cost of supervision: the higher the cost, the lower the level of supervision.

(2) Medium profit gap

When the profit of medical overuse is at a medium level and the supervision cost is at a low level, NHSA naturally tends to supervise loosely and medical institutions tend to gain profit in such a low-risk regulatory environment, whereas when the supervision cost is low, the strategy is mixed.

(3) Low profit gap

When the profits of medical overuse are low enough, medical institutions will choose appropriate medical use regardless of NHSA's loose supervision. This indicates that without the motivation of profit, medical institutions will naturally promote appropriate medical use. Meanwhile, the medical institutions' strategy also affects NHSA's decisions. In such a scenario, regulatory measures are unnecessary. Therefore, even when the supervision cost changes, NHSA will still choose loose supervision. Under this condition, the strategic choice of both sides reaches the ideal state of medical supervision, i.e., to supervise without exertion.

## 4. Simulation Analysis

### 4.1. Evolutionary Simulation of the Game System

Based on the analysis above, we can obtain the evolutionary game results between NHSA and medical institutions under various scenarios, but the analysis does not explain how to achieve these results. We will use MATLAB as an analysis tool to simulate the dynamic evolution of the strategies of NHSA and medical institutions.

Our research is mainly based on the background of China's medical insurance payment method, fee-for-service. We have conducted surveys in medical insurance bureaus in many cities in southwest China and summarised four kinds of scenarios as below. These situations can represent the reality of the regulation of NHSA in China. Through simulation with parameters under different scenarios, we can provide reference opinions for policy-makers.

In this section, six simulation experiments are conducted to explore the dynamic evolution of the strategies, as shown in Figure 1. According to the results, we can divide all scenarios into four kinds.

1. Profit gap at low level and supervision cost at any level

For Scenario 1 and Scenario 4, the unique ESS under the two situations is the same (0,1). As the profit gap between medical overuse and appropriate medical use is not large enough, hospitals will always choose the “appropriate medical use” strategy. At this time, no matter how high the cost that NHSA needs to pay, it will choose the “loose supervision” policy.

(2) Profit gap at medium and high level and supervision cost at high level

For Scenario 2 and Scenario 3, (0,0) is the ESS. In both cases, NHSA will pay a high cost for governing strictly so that “loose supervision” is the behaviour strategy. Naturally, with no limitation on regulation and considerable profits brought by medical overuse, these medical institutions will engage in medical overuse.

(3) Profit gap at high level and supervision cost at low level

Under Scenario 6, the ESS is (1,0). The low cost of strict supervision drives NHSA to supervise strictly, while the high profits brought by medical overuse make the hospitals choose to treat excessively.

(4) Profit gap at medium level and supervision cost at low level

Specifically, there is no ESS for Scenario 5. At this time, increasing the profit gap will drive the system to evolve to (1,0). Decreasing the profit gap will drive the system to evolve to (0,1). Increasing the supervision cost will drive the system to evolve to (0,0).

### 4.2. Numerical Simulation of Stability Influencing Factors

In the real world, hospitals are always driven to engage in medical overuse by the high profit gap, and with the limitations of high supervision costs, administration's supervision is mainly cursory and infrequent. Comparatively, the hypothesis of Scenario 6 is more consistent with the real world. Second, specifically, there is no ESS in Scenario 5. Therefore, we will conduct some numerical experiments for further analysis. The following simulation analysis background is used to set the relevant parameters to meet the conditions corresponding to Scenario 5 and Scenario 6. The data of the parameters setting, as shown in Tables 6 and 7, is first collected from field survey on medical institutions and local Healthcare Security Administration in southwestern China. The data is private and not allowed to be released to public. Via expert interviews method, we get a rough ratio of several costs and profits involved in the research and then we processed the rough data collected according to the model.

#### 4.2.1. Impact of Initial Intentions on Evolution in Scenario 5

We will analyse the evolution trend of Scenario 5 for further understanding. Based on the actual situation, the initial parameters are set in Table 6.

First, it is not difficult to realise that the behaviour of the participants is cyclical and there is no stable strategy. As can be seen from Figure 2, the preferences of NHSA and the medical institutions are not clear. No matter what the initial status is, the proportion of strategic choice between the two sides fluctuates a little, and the medical institutions always tend to adopt appropriate medical use at the beginning.

When the likelihood of NHSA choosing “strict supervision” as the initial strategy is higher, the fluctuation cycle of medical institutions' strategy choice is longer. Similarly, the larger the proportion of medical institutions choosing the initial strategy of “medical overuse,” the longer the fluctuation cycle of NHSA's strategy choice.

#### 4.2.2. Impact of Profit and Cost on Evolution in Scenario 5

Next, we conduct several numerical experiments to derive the impacts of parameters on the evolutionary results. We fix other parameters and conduct experiments when Δ*R* = 46, 56, 66, and 76 and *C*_1_ = 5, 10, 15, and 25. All initial probabilities *p* = *q* = 0.5. The dashed line represents the evolution process when the parameters change, and the solid line represents the original evolution process of both sides.

The increase of the profit gap Δ*R* will shorten the evolutionary cycle, as shown in Figure 3. With the increase of supervision cost *C*_1_, the evolutionary cycle of the game gets longer, and then, it gets shorter after reaching a particular value, as shown in Figure 4.

Specifically, when Δ*R* reaches a certain value, the strategy of NHSA will change from “loose” to “strict,” and the strategy of medical institutions will change from “appropriate medical use” to “medical overuse.” It is worth noting that the increase of *C*_1_ will ultimately make medical institutions adopt “medical overuse” as their policy.

#### 4.2.3. Impact of Profit, Cost, and Probability of Complaint on Evolution in Scenario 6

To better understand the evolution of Scenario 6, we analyse the impacts of three parameters on the evolutionary results separately, including the supervision cost *C*_1_, the profit gap Δ*R*, and the probability of patients' complaints, *θ*.

Based on the actual situation, the initial parameters are set in Table 7.

The first experiments are conducted when Δ*R* = 66, 86, 106, and 126. The second experiment is conducted when *C*_1_ = 0, 8, 16, and 24. The third experiment is conducted when *θ* = 0.1, 0.3, 0.5, and 0.7. For all experiments, the initial probabilities *p* = *q* = 0.5.

Similar to the analysis above, the dashed line represents the evolution process when the parameters change, and the solid line represents the original evolution process of both sides. As is shown in Figure 5, with the increase of the profit gap, the convergence speed of NHSA becomes slightly slow. Conversely, the convergence speed of medical institutions becomes fast clearly with the profit gap increasing. The result shows that the excessive profit gap brought by medical overuse is a main contributor for hospitals to engage in medical overuse, but not a key impact factor of NHSA's strategy choice.

As shown in Figure 6, the convergence rate of the medical institution's strategy increases with the increase of supervision cost. However, the change of supervision cost has little effect on the strategy choice of the medical institution. By contrast, the convergence rate of NHSA's strategy decreases heavily with the increase of supervision cost. When *C*_1_ = 24, the tendency of NHSA's strategy drops to a certain degree but then rises and converges to the ESS. The result shows that the higher the supervision cost, the lower the willingness of NHSA to supervise strictly, and when the cost reaches a particular value, NHSA will finally choose “loose supervision.”

As shown in Figure 7, the convergence rate of both sides' strategies decreases with the increase of the probability of patients questioning and complaining. The more likely patients are to report, the more cautious medical institutions are, so that the less likely they are to adopt medical overuse. However, the more likely patients are to report, the more likely NHSA is to rely on patients' supervision, and the less it is involved in supervision.

## 5. Conclusions

This study starts from bounded rationality, builds an evolutionary game model to study the relations between the NHSA and medical institutions, and reveals the dynamic evolution process between the supervision of NHSA and medical overuse of medical institutions. By analysing the evolutionary stable strategies, numerical studies are conducted and show good results. Through the numerical simulation and sensitive experiments under various scenarios, we obtain the following results:

1. In the most common situation that the profit gap is at a medium level, the regulatory measures of NHSA work well. Medical institutions' strategies change as the supervision cost changes. When the supervision cost is high, medical institutions tend to choose medical overuse, otherwise choose appropriate medical use
2. In the other two scenarios, regulatory measures of NHSA cannot work: if the profit gap is too high, the medical institution will definitely choose medical overuse. While if the profit gap is lower than the fines and reputation loss caused by medical overuse, the medical institution will choose appropriate medical use no matter a punishment mechanism is set or not
3. Patient involvement in supervision exerted a significant impact on the strategies of medical institutions and NHSA. The more likely patients are to report, the less possibility NHSA is involved in supervision, and the less likely medical institutions are to adopt medical overuse

From the results of the study, we know that NHSA should strengthen supervision and issue relevant policies to curb behaviours such as prescribing excess drugs and medical tests. And NHSA should also improve the public's participation in health regulation. Multiple participation and supervision are key to preventing excessive diagnosis and treatment. To decrease medical overuse and rationalise hospital costs, supervision of hospitals by NHSA is essential. More research in this area is urgently needed. Specifically, we obtain some management insights as follows:

1. It is necessary to establish a comprehensive medical insurance payment system to curb excessive medical use and promote reasonable medical examination and treatment
2. The authorities should consider how to reduce the cost of supervision by optimising the process systematically. In this manner, NHSA would supervise frequently so that the probability of medical overuse can be reduced
3. Some activities on education of medical knowledge for the public should be carried out to enhance the awareness of the patients' cognitive status on excessive medical examination and treatment. NHSA should try its best to facilitate the supervision of the public through multiple channels

There are two potential directions that could be investigated in the future. First, since the supervision of the medical overuse involves patients, also considering patients as stakeholders and modelling as tripartite game can be studied. Second, as there are many different hospitals and institutions, competition and cooperation among medical institutions can be included.

## Figures and Tables

**Figure 1:** The evolutionary processes of six scenarios.

**Figure 2:** Evolution results of Scenario 5 under different behaviour ratios.

**Figure 3:** Evolution process of Scenario 5 under different Δ*R* values.

**Figure 4:** Evolution process of Scenario 5 under different *C*_1_ values.

**Figure 5:** Evolution process of Scenario 6 under different Δ*R* values.

**Figure 6:** Evolution process of Scenario 6 under different *C*_1_ values.

**Figure 7:** Evolution process of Scenario 6 under different *θ* values.

**Table 1:** Parameter symbol descriptions in the evolutionary game.

Stakeholders	Parameters	Descriptions
Medical institutions	*R*_1_	Revenue of appropriate medical use
	*R*_2_	Revenue of medical overuse
	*R*_3_	Revenue of reputation given by NHSA because of appropriate medical use
	*F*	Penalty from NHSA because of medical overuse behaviour discovered
	*M*	Reputation loss because of medical overuse behaviour discovered such as decreased credibility and reduced number of patients
	*θ*	Probability of patients questioning and complaining about medical institutions' medical overuse
	*q*	Probability of medical institutions adopting appropriate medical use
NHSA	*C*_1_	All the costs of NHSA offering strict supervision
	*C*_2_	Cost and loss to NHSA's verification behaviour because of medical overuse behaviour complained by patients, mainly including: verification cost, credibility decline, and reputation loss
	*p*	Probability of NHSA offering strict supervision

**Table 2:** The payoff matrix of the model.

		Medical institutions	
		Appropriate medical use (*q*)	Medical overuse (1 − *q*)
NHSA	Strict supervision (*p*)	−*C*_1_, *R*_1_ + *R*_3_	−*C*_1_ + *F*, *R*_2_ − *F* − *M*
	Loose supervision (1 − *p*)	0, *R*_1_	*θ*(*F* − *C*_2_), *R*_2_ − *θ*(*F* + *M*)

**Table 3:** The det *J* and trac *J* at each LEP.

LEP	det *J*	trac *J*
(0,0)	[(1 − *θ*)*F* + *θC*_2_ − *C*_1_][*R*_1_ − *R*_2_ + *θ*(*F* + *M*)]	*F* − *θC*_2_ − *C*_1_ + *R*_1_ − *R*_2_ + *θM*
(0,1)	*C*_1_[*R*_1_ − *R*_2_ + *θ*(*F* + *M*)]	−[*R*_1_ − *R*_2_ + *θ*(*F* + *M*) + *C*_1_]
(1,0)	−[(1 − *θ*)*F* + *θC*_2_ − *C*_1_](*R*_1_ − *R*_2_ + *R*_3_ + *F* + *M*)	*R*_1_ − *R*_2_ + *R*_3_ + *M* − *θF* − *θC*_2_
(1,1)	−(*R*_1_ − *R*_2_ + *R*_3_ + *F* + *M*)*C*_1_	*C*_1_ − (*R*_1_ − *R*_2_ + *R*_3_ + *F* + *M*)
(*p*^∗^,*q*^∗^)	-AB	0

Note: AB denotes ((*R*_1_ − *R*_2_ + *R*_3_ + *F* + *M*)∗[*R*_1_ − *R*_2_ + *θ*(*F* + *M*)])/(*R*_3_ + (1 − *θ*)(*F* + *M*))∗(*C*_1_[(1 − *θ*)*F* + *θC*_2_ − *C*_1_])/((1 − *θ*)*F* + *θC*_2_).

**Table 4:** The evolutionary stability of each LEP.

Scenarios	LEP	det *J*	trac *J*	State
Scenario 1: *R*_1_ − *R*_2_ < *θ*(*F* + *M*) *C*_1_ > (1 + *θ*)*F* + *θC*_2_	(0,0)	—	Uncertain	Saddle point
	(0,1)	+	—	ESS
	(1,0)	+	+	Unstable
	(1,1)	—	Uncertain	Saddle point
Scenario 2: *θ*(*F* + *M*) < *R*_2_ − *R*_1_ < *R*_3_ + *F* + *M* *C*_1_ > (1 + *θ*)*F* + *θC*_2_	(0,0)	+	—	ESS
	(0,1)	—	Uncertain	Saddle point
	(1,0)	+	+	Unstable
	(1,1)	—	Uncertain	Saddle point
Scenario 3: *R*_2_ − *R*_1_ > *R*_3_ + *F* + *M*, *C*_1_ > (1 + *θ*)*F* + *θC*_2_	(0,0)	+	—	ESS
	(0,1)	—	Uncertain	Saddle point
	(1,0)	—	Uncertain	Saddle point
	(1,1)	+	+	Unstable
Scenario 4: *R*_2_ − *R*_1_ < *θ*(*F* + *M*), *C*_1_ < (1 + *θ*)*F* + *θC*_2_	(0,0)	+	+	Unstable
	(0,1)	+	—	ESS
	(1,0)	—	Uncertain	Saddle point
	(1,1)	—	Uncertain	Saddle point
Scenario 5: *θ*(*F* + *M*) < *R*_2_ − *R*_1_ < *R*_3_ + *F* + *M* *C*_1_ < (1 + *θ*)*F* + *θC*_2_	(0,0)	—	Uncertain	Saddle point
	(0,1)	—	Uncertain	Saddle point
	(1,0)	—	Uncertain	Saddle point
	(1,1)	—	Uncertain	Saddle point
	(*p*^∗^,*q*^∗^)	+	0	Central point
Scenario 6: *R*_2_ − *R*_1_ > *R*_3_ + *F* + *M* *C*_1_ < (1 + *θ*)*F* + *θC*_2_	(0,0)	—	Uncertain	Saddle point
	(0,1)	—	Uncertain	Saddle point
	(1,0)	+	—	ESS
	(1,1)	+	+	Unstable

**Table 5:** Relationship between ESS and levels of profit gap and supervision cost.

Level of profit gap	Level of supervision cost	Equilibrium stable strategies	
		NHSA	Medical institutions
High	High	Loose supervision	Medical overuse
	Low	Strict supervision	Medical overuse
Medium	High	Loose supervision	Medical overuse
	Low	—	—
Low	High	Loose supervision	Appropriate medical use
	Low	Loose supervision	Appropriate medical use

**Table 6:** Initial parameters setting in Scenario 5.

Parameters	*R*_1_	*R*_2_	*R*_3_	*F*	*M*	*C*_2_	*θ*	*C*_1_
Scenario 5	90	140	20	40	35	20	0.6	20

**Table 7:** Initial parameter setting in Scenario 6.

Parameters	*R*_1_	*R*_2_	*R*_3_	*F*	*M*	*C*_2_	*θ*	*C*_1_
Scenario 6	80	150	10	40	15	20	0.6	5

## Data Availability

No data were used to support this study.
